The article "Bacterial Transmembrane Proteins that Lack N-Terminal Signal Sequences" was published in 2011. Journal: PLoS One.

# Bacterial Transmembrane Proteins that Lack N-Terminal Signal Sequences

**DOI:** 10.1371/journal.pone.0019421

**Published:** 2011-05-04

**Authors:** Arryn Craney, Kapil Tahlan, David Andrews, Justin Nodwell

**Affiliations:** Department of Biochemistry and Biomedical Sciences, McMaster University, Hamilton, Ontario, Canada; The Scripps Research Institute, United States of America

## Abstract

Tail-anchored membrane proteins (TAMPs), a class of proteins characterized by their lack of N-terminal signal sequence and Sec-independent membrane targeting, play critical roles in apoptosis, vesicle trafficking and other vital processes in eukaryotic organisms. Until recently, this class of membrane proteins has been unknown in bacteria. Here we present the results of bioinformatic analysis revealing proteins that are superficially similar to eukaryotic TAMPs in the bacterium *Streptomyces coelicolor*. We demonstrate that at least four of these proteins are bona fide membrane-spanning proteins capable of targeting to the membrane in the absence of their N-terminus and the C-terminal membrane-spanning domain is sufficient for membrane targeting. Several of these proteins, including a serine/threonine kinase and the SecE component of the Sec translocon, are widely conserved in bacteria.

## Introduction

Protein translocation into and across the lipid bilayer is an essential process in all kingdoms of life. Most proteins are inserted into the membrane by the well-conserved Sec pathway, consisting of a membrane-spanning translocase SecYEG in bacteria and Sec61 in eukaryotes. Many accessory proteins aid in protein targeting and insertion, including in particular the signal recognition particle (SRP), and its cognate membrane receptor [1], [2]. To be targeted to the membrane via the Sec system, a protein must have an N-terminal signal sequence for recognition by the SRP. Signal sequences are typically 20–30 amino acids long and consist of an N-terminal domain with one or more positively charged amino acids, followed by an H-domain of 8–12 hydrophobic residues and, for proteins that are secreted, a C-domain recognition site for peptide cleavage [3]. During co-translational targeting the signal sequence is recognized and bound by the SRP as the N-terminus of the nascent polypeptide emerges from the ribosome. The ribosome/nascent peptide are then brought to the membrane for insertion through an interaction with the SRP receptor FtsY [4] and transferred to the SecYEG translocon for insertion [5]. (For reviews of Sec translocation see [3], [6], [7], [8], [9], [10].

While the majority of membrane proteins are targeted to the membrane via Signal sequence/Sec translocon-dependent mechanisms, another system has been identified in eukaryotes for targeting tail anchor membrane proteins (TAMPs) [11], [12]. Eukaryote TAMPs carry out a wide range of biological functions, many of which involve membranes. Examples include the Bcl-2 protein, a major player in the apoptosis pathway, the SNARE proteins which are involved in vesicle targeting and fusion, and the Sec61β protein, which is a component of the eukaryotic Sec translocon [13], [14]. Bcl-2, the SNAREs and Sec61β all lack the N-terminal signal sequence required for SRP-targeting and are instead targeted to the membrane via a single C-terminal transmembrane domain, the tail anchor.

The article "Bacterial Transmembrane Proteins that Lack N-Terminal Signal Sequences" was published in 2011. Journal: PLoS One.

All of the TAMPs that have been investigated biochemically to date are found in eukaryotes. Recently however, a bioinformatic approach was used to demonstrate the existence of TAMP-like proteins in the Gram-negative bacteria *Escherichia coli* and *Rickettsia prowazekii* as well as the archeon *Methanococcus maripaludis* [15]. This work suggests that in fact, tail-anchored membrane proteins are universal and that they make up similar proportions of all proteomes [15]. Our work adds to this, providing experimental evidence of these bacterial tail anchor membrane proteins. We have taken advantage of a newly developed algorithm, TAMP finder (Brito et al., Manuscript in Preparation) to identify membrane-proteins encoded in the Gram-positive bacterium *Streptomyces coelicolor*. Similarly, we find a large number of proteins that are superficially similar to the eukaryotic TAMPs in that they lack signal sequences and contain single C-terminally located transmembrane domains. We have used several biochemical approaches to test these predictions and find that indeed, many of these proteins are transmembrane proteins and that the tail sequences are sufficient for membrane targeting. These include important proteins including the SecE component of the translocon and members of the bacterial serine/threonine (ser/thr) protein kinase family.

## Results

### Putative membrane proteins lacking signal sequences and exhibiting broad conservation in prokaryotes

A genome-wide search using the “TAMP finder” program (Brito et al., Manuscript in Preparation) identified 73 putative tail-anchor membrane proteins (TAMPs) in *Streptomyces coelicolor*. This program was designed to identify TAMPs encoded in eukaryotic genomes by seeking polypeptide sequences having the known TAMP properties. These include a putative C-terminally located transmembrane domain, the tail anchor, and the absence of an obvious N-terminal signal sequence. To further test these candidates, we analyzed each of them individually using the transmembrane prediction program TMHMM [16]. We restricted subsequent analysis to those proteins having one or, in a few cases two, strongly-predicted transmembrane domains near the C-terminus. We then used SignalP, a program that predicts SRP signal sequences, and visual inspection to further confirm that these proteins lack candidate N-terminal signal sequences [17]. 20 of the 73 predicted polypeptides identified by TAMP finder met both criteria (Table 1 and Figure 1). During this analysis, careful consideration was taken in scanning the upstream regions of the predicted translational start site to ensure proteins were not mis-annotated. Those with mis-annotated start sites that contained N-terminal signal sequences were removed from the analysis.

The article "Bacterial Transmembrane Proteins that Lack N-Terminal Signal Sequences" was published in 2011. Journal: PLoS One.

**Figure 1:** Putative bacterial membrane proteins lacking N-terminal Signal Sequences. (**A**) The N-terminal sequences of five strongly predicted *S. coelicolor* transmembrane proteins (FtsY, SCO0041, SCO1101, SCO1374 and SCO2176) are shown, illustrating their high hydrophobicity and correspondingly low hydrophilicity. Hydrophobic residues are shaded grey. Double arginine residues are bolded. (**B**) The N-terminal sequences of the *S. coelicolor* cytoplasmic protein (ActR) and (**C**) 20 predicted tail anchor membrane proteins lacking obvious signal sequences are shown to illustrate their highly hydrophilic N-terminus.

**Table 1:** Highest Confidence *S. coelicolor* Tail Anchor Membrane Proteins.

Protein	Size(aa)	Proposed Function	N-terminus	Tail Anchor	Homologues
SCO1166	110	hypothetical	out	AAGLILLIWLPWWAALLIVLGVPAAAYLTLDPSQRRRLRRVSRKEIGR	streptomycete
SCO1431	80	hypothetical	Out	PKILEHVLGWTLVVVVAMLVVQLGLL	streptomycete
SCO2124 *	205	hypothetical	In	WLTTLSIGGFLGGFATLVVRMRTGDEDDDDPGRGAVV	actinomycete
SCO2199	89	hypothetical	Out	VGSRRRSSWVSTVVVLGCVAAVIVLLGYLNFRAPY	streptomycete
SCO2900	110	hypothetical	out	TGAPRMERVVPVALVVAGVVGLLALGGTRRRKR	actinomycete
SCO2973	417	Ser/Thr Kinase (PkaB)	In	RRRRIAVGAGAVALVAAIGVGTWLATGGDEDGGGPQDTRNSAPAAP	actinomycete
SCO3544 *	132	hypothetical	In	PVALGVSPVASATVASVAAVVALGLGAWCLTQV	actinomycete
SCO3860	576	Ser/Thr Kinase	In	RRRRRPGPPARVALPVLLLALACYAVGFWALTRI	streptomycete
SCO4008	192	TetR-like	In	APDLLFLLVAMANWAVVVPQMKRILVGGGDAGTDGLRDSIKKAARRIVDR	actinomycete
SCO4033	96	hypothetical	In	AASSGPRVGLIVGIVAAVIVVAAVAWLALG	streptomycete
SCO4174	83	hypothetical	In	HKARSRRRAGLDGATVSGLLTVLCVATLLVTITFAV	*S. lividans*
SCO4646	94	SecE	In	SRNQLTTYTTVVIIFVVIMIGLVTLIDYGFSHAAKYVFG	Most bacteria
SCO4959	85	hypothetical	In	TAARRLMWLLLGAAAVAFTVWALTVQPWVEPPSETTPPVTGWEGWS	streptomycete
SCO5157 *	317	CorA	In	DYMPETHWKFGYPLVLSVTVCICLGIHRTLKRNGWL	Most bacteria
SCO5344 *	107	SpdD2	In	GGGTAVVLVVGAVLVSMLLAVAITAASVAVCAVVLRSLLASDAKRR	streptomycete
SCO6904	336	hypothetical	Out	GADATLWLIGGAAVLIAAGGGALAVARRSRTDSHTQDNTGS	streptomycete
SCO7096	114	hypothetical	In	RRYARLRRMSRVALAVLAATVMVLLVALVLVAAG	streptomycete
SCO7133	113	hypothetical	In	RGTMIAMTAIGLTIFVCTAVVVGSMT	streptomycete
SCO7199	131	hypothetical	In	RRLGRILAGAAALAVLLGLFTCLPEEPPGLPTGPEDTSPPRTSSAVVES	streptomycete
SCO7330	78	hypothetical	Out	GWAKGPMALILAVVVIFAVGLLGYALALIY	actinomycete

*denotes 2 predicted transmembrane domains at the C-terminus.

The article "Bacterial Transmembrane Proteins that Lack N-Terminal Signal Sequences" was published in 2011. Journal: PLoS One.

Putative signal sequences at the N-termini of the *S. coelicolor* FtsY and four other proteins annotated as membrane proteins are shown in Figure 1. All have stretches of 8–10 hydrophobic residues: these are the predicted binding sites of the SRP [3]. In contrast, the known cytoplasmic protein ActR has a hydrophilic N-terminus. Similarly, the 20 candidates listed below ActR, with the exception of SCO6904, also have largely hydrophilic N-termini (Figure 1). These proteins therefore lack obvious N-terminal signal sequences. The ‘twin-arginine repeat’ or TAT pathway is involved in the secretion of folded proteins and has not been implicated in membrane insertion [18]. We note however that these candidates also lack the characteristic Z-R-R-ϕ-X-X (where Z is a polar residues, X-X are hydrophobic residues and ϕ is any residue) although SCO4033 has two arginines embedded in the N-terminal sequence A**RR**PRTWAALA. It is unlikely that this could serve as a target for TAT-mediated secretion.

The 20 candidates in Table 1 represent a wide range of important biological functions. These include a conspicuous number of hypothetical membrane proteins of less than 100 amino acids (SCO1431, SCO2199, SCO4033, SCO4174, SCO4959 and SCO7330), two serine/threonine protein kinases (SCO2973 and SCO3860), the SecE component of the Sec translocon (SCO4646) proposed to be a tail-anchored membrane protein in many organisms, including *Archea* [15], a CorA-like Mg^2+^ transporter (SCO5157) [19] and the SpdD2 protein believed to be involved in transfer of plasmid DNA in streptomycetes (SCO5344) [20], [21]. Many of these proteins are highly conserved in the actinomycetes and two are conserved generally in prokaryotes [15], [19] (Table 1). While, the majority of these proteins are predicted to have a topology with the N-terminus facing into the cell, several are predicted to have their N-termini projecting out of the cell (Table 1).

While a large number of these proteins are small hypothetical proteins, we are confident that these represent expressed genes rather than artefacts of genome annotation. Only membrane proteins conserved in multiple streptomycetes and possible having orthologues in other actinomycetes were included in our analysis. For example, SCO2900 is predicted to encode a 110 residue polypeptide that is conserved within the Streptomycetes and related Actinomycetes (Figure 2a). Conserved features of this protein include 3 absolutely conserved residues (P29 R34 P37 with respect to the *S. coelicolor* protein sequence) and the C-terminal transmembrane domain followed by a small stretch of 4 positively charged residues, suggesting an N-terminus “out” orientation. Sequences from related Actinomycetes were found to contain an approximately 30 residue deletion upstream of the predicted tail anchor and there is a small C-terminal extension in *Corynebacterium* proteins. SCO7133-like proteins were found in some Streptomycetes, and in no other genera (Figure 2b). Although a C-terminal transmembrane domain is consistently predicted among SCO7133 paralogues, the amino acid identity in this domain is low. Four positively charged residues are located directly upstream of the transmembrane domain, suggesting the N-terminus of this protein is facing into the cell. This predicted topology was shared among the SCO7133-like paralogues. The large N-terminal extension predicted in *S. lividans* TK24 is most likely mis-identification of the start site; regardless, this extended region does not contain an N-terminal signal sequence.

The article "Bacterial Transmembrane Proteins that Lack N-Terminal Signal Sequences" was published in 2011. Journal: PLoS One.

**Figure 2:** Alignments of predicted tail-anchor membrane proteins. (**A**) SCO2900 from *S. coelicolor* aligned with various orthologues from other streptomycetes and actinomycetes (**B**) SCO7133 from *S. coelicolor* aligned with various orthologues from other streptomycetes. The *S. lividans* extended leader sequence is MGRHRPREDRRPTGTAPTAAPRH. Absolutely conserved residues are shaded black and marked with *, similar residues are shaded grey. Possible topology predicting residues are marked with+and the C-terminal transmembrane domains are boxed and shaded grey.

### Four integral membrane proteins

We chose 5 of the candidates in Table 1 to test the prediction that they are integral membrane proteins: two small hypothetical proteins (SCO2900 and SCO7133), the ser/thr kinase PkaB (SCO2973), SecE (SCO4646) and a predicted TetR-like transcription factor (SCO4008). The known cytoplasmic protein ActR served as a control. All six proteins were expressed in *S. coelicolor* under the thiostrepton-inducible promoter *tipA* such that they had an N-terminal FLAG-tag for visualization by Western analysis.

Protoplasts of cells expressing these proteins were isolated from lysozyme-treated cells. The protoplasts were subsequently lysed, fractionated by ultracentrifugation and the pellets and supernatants analyzed by Western analysis with anti-FLAG antibodies. As expected, ActR was found exclusively in the supernatant (Figure 3a). Similarly, in spite of having a predicted transmembrane domain, SCO4008 was found exclusively in the supernatant, consistent with its probable role as a DNA binding transcription factor. The other four proteins were contained exclusively in the pellets.

The article "Bacterial Transmembrane Proteins that Lack N-Terminal Signal Sequences" was published in 2011. Journal: PLoS One.

**Figure 3:** Membrane-association of five candidates. (**A**) Cells were fractionated into pellet (P) and supernatant (S) fractions and Western blot analysis directed against the FLAG epitope was used to determine the localization of the putative membrane proteins SCO2900, SCO2973, SCO4008, SCO4646 and SCO7133. ActR was used as a cytoplasmic control. (**B**) The pellets from (A) were subjected to sucrose gradient ultracentrifugation and 1 ml fractions were collected with fraction 1 corresponding to the highest density and fraction 10 the lowest. Fractions 2 to 4 (underlined) correspond to sedimentation profiles of known membrane proteins. (**C**) Carbonate extraction of TAMP proteins. Cell lysate was mixed with either sucrose (−) or carbonate (+) and separated into pellet (P) and supernatant (S) fractions. Fractions were subjected to Western blot analysis. The peripheral membrane protein RamC was used as a control.

To determine whether the pellet-associated proteins SCO2900, PkaB, SecE or SCO7133 were membrane-associated, the pellets from this centrifugation step were subjected to sucrose gradient ultracentrifugation. To locate the membrane fractions we used antibodies against the known Sec-dependent transmembrane protein, SecG for Western analysis. Consistent with previous analysis of membrane-proteins using this procedure SecG was found primarily in the 2^nd^ and 3^rd^ fractions (Figure 3b) [22]. Consistent with membrane association, SCO2900, SCO2973 (PkaB), SCO4646 (SecE), and SCO7133 were also found predominantly in fraction 2 and 3. None were found in the pellet (Figure 3b) as would be the case if these proteins were simply insoluble hydrophobic inclusions.

Extraction of the membranes at pH 11.4 using sodium carbonate was then used to distinguish between proteins that were peripherally or integrally associated with the membrane [23]. Cells expressing the four candidates demonstrated above to be membrane-associated (Figure 3a and b) were converted to protoplasts, lysed, subjected to carbonate extraction and then fractionated into membrane-containing (P) and cytosolic (S) fractions. As shown in Figure 2c, SCO2900, SCO2973 (PkaB) and SCO4646 (SecE) remained entirely in the membrane-containing fraction. Some SCO7133, possibly 30% of the total, was found in the supernatant fractions in this particular experiment. We suspect that this is a result of prolonged induction of the *tipA* promoter that drives expression of the fusion. Importantly, only a very modest amount of protein was moved from the pellet to the supernatant after carbonate extraction. In contrast, the protein RamC, which we have shown previously to be membrane-associated via interactions with other proteins [24], was almost completely separated from the membranes by treatment with sodium carbonate. This is striking because RamC is an extremely hydrophobic protein and yet could still be rendered soluble in this way. This strongly suggests that the other four proteins remained in the pellet fractions because they are integral membrane proteins.

The article "Bacterial Transmembrane Proteins that Lack N-Terminal Signal Sequences" was published in 2011. Journal: PLoS One.

### Tail sequences are sufficient for membrane targeting

To investigate whether the tail sequences of these proteins are sufficient for membrane targeting, the C-terminal sequences of three candidates, SCO2973 (PkaB), SCO4646 (SecE) and SCO7133 (including 11 amino acid residues upstream of the putative transmembrane domain, see materials and methods) were fused to the cytoplasmic protein eGFP generating eGFP-2973, eGFP-4646 and eGFP-7133. SCO2900 was not included for analysis as its N-terminus is predicted to face out of the cell. Again, these fusions were expressed in *S. coelicolor* using thiostrepton; protoplasts prepared and lysed then fractionated using ultracentrifugation. Fractions containing the fusions were then identified using Western analysis with anti-GFP antibodies. Cross-reactive bands to the eGFP antibody are visible with the eGFP-7133 fusion protein, these bands are also present in the other samples; however, they are not contained in the field of the image. As expected, the unfused eGFP protein was contained entirely in the supernatant (Figure 4). In contrast, all fusions to eGFP were found completely in the pellet fractions (Figure 4).

**Figure 4:** Localization of eGFP tail anchor fusions. Putative tail anchor transmembrane domains from SCO2973, SCO4646 and SCO7133 were fused to the C-terminus of the cytoplasmic protein eGFP and localization to the pellet (P) and supernatant (S) fractions was determined in the presence of either sucrose (−) or carbonate (+). Unfused eGFP is shown for comparison. Localization was detected by Western blot analysis against eGFP.

The three eGFP-tail sequence fusions were subjected to carbonate extraction to determine whether they behaved as integral membrane proteins. All three proteins remained in the pellet fraction regardless of the treatment with sodium carbonate, suggesting that they were integral membrane proteins (Figure 4). The ability of the transmembrane domain from the three tail-anchor proteins to relocate eGFP to the pellet and resist carbonate extraction strongly suggests that all information required for targeting to the membrane is found in the C-termini of these proteins.

The article "Bacterial Transmembrane Proteins that Lack N-Terminal Signal Sequences" was published in 2011. Journal: PLoS One.

### Bacterial Tail Anchor Membrane Proteins are capable of facing into and out of the cell

During the topology prediction, we noted that while the majority of our putative TAMPs were predicted on the basis of the ‘positive charge in’ rule [25] to have their N-termini face into the cell, 6 of the 20 were predicted to have their N-termini exterior to the cell, in contrast to the eukaryote paradigm. In order to test this we subjected the 4 candidates (SCO2900, SCO2973, SCO4646 and SCO7133) to Proteinase K digestion with ActR, a cytoplasmic protein, serving as a control for cell lysis (Figure 5). We found that with high doses of proteinase, all of the fusions were rapidly degraded to the point where they were undetectable by anti-FLAG tag Western analysis (data not shown). At lower proteinase concentrations however, including those shown in Figure 5, SCO2900 was consistently more sensitive to proteinase digestion than SCO2973, SCO4646 or SCO7133, suggesting this proteins FLAG-tag is external to the cell, along with the bulk of the protein, and that it is therefore susceptible to proteolytic removal. We take this as evidence that while the N-termini of SCO2973, SCO4646 and SCO7133 are intracellular, SCO2900 may project it's N-terminus out of the cell, as predicted by the ‘positive charge in’ rule [25].

**Figure 5:** Protease protection assay to assess TAMP orientation at the membrane. Protoplasts expressing ActR, SCO2900, SCO2973, SCO4646 and SCO7133 were subjected to increasing concentration of Proteinase K (PK). Exterior facing N-termini were expected to be susceptible to Proteinase K digestion; while inward facing N-termini were expected to be protected. Visualization of the extent of degradation was detected by Western blot analysis against the FLAG epitope.

## Discussion

We have identified a previously uncharacterized class of bacterial membrane proteins in *S. coelicolor* that lack the N-terminal signal sequences and, rather, depend on C-terminal transmembrane domains for membrane targeting. This is the first time such an observation has been biochemically demonstrated in a prokaryote. Aside from their C-terminal sequences, these proteins do not appear to contain any additional sequence motif for membrane targeting as the C-termini alone from three of these proteins can render eGFP entirely membrane-associated (Figure 4). Furthermore, the remarkable diversity of the N-terminal domains of these proteins, which exhibit no universally conserved sequence characteristics, strongly argues for a membrane targeting mechanism that depends primarily, if not entirely on, the C-terminal domains.

The article "Bacterial Transmembrane Proteins that Lack N-Terminal Signal Sequences" was published in 2011. Journal: PLoS One.

Among the candidates that we have worked with here are at least two known proteins of considerable interest, PkaB (SCO2973), one of the so-called “eukaryotic” ser/thr protein kinases found in streptomycetes and other prokaryotes, and SecE from the Sec translocon. Orthologues of these proteins have been investigated in several bacteria previously; however, to our knowledge the possible tail-anchoring is a new observation [26], [27], [28].

While little is known about PkaB in *S. coelicolor*, it is closely related to the *Mycobacterium tuberculosis* protein kinase PknA. The *pknA*_TB_ gene is adjacent to a second ser/thr kinase gene *pknB*_TB_, (unfortunately referred to as *pkaA* in *S. coelicolor*. These two Mycobacterial kinases have been implicated in cell division and the maintenance of cell shape and it has been suggested that they may phosphorylate components (FtsZ and FipA) of the division apparatus [29]. The single C-terminal transmembrane domain has been previously noted; however, the absence of N-terminal signal sequences was not. The importance of PknA in *M. tuberculosis* suggests, that understanding the mechanism with which this kinase targets to the membrane could lead to new drug targets for combating this pathogenic bacteria.

SecE is similarly a highly studied and important protein. Its role in secretion is to aid in forming the protein conducting channel, the SecYEG translocase, by stabilizing SecY and by contributing residues to the active centre in the translocase [5], [30]. The *E. coli* SecE protein, arguably the best studied prokaryotic example, is a 127 amino acid, Sec-dependent polytopic transmembrane protein having three transmembrane sequences. In contrast, the *S. coelicolor* orthologue that we have investigated, SCO4646, is a 79 amino acid protein having a single transmembrane domain at its C-terminus: we confirmed that this characterization is not due to a mis-identification of the open reading frame's 5′ end. These results are also in agreement with recently published bioinformatic data from the SecE of *M. maripaludis* [15].

The eukaryotic orthologues of SecE, Sec61β, are also well-known tail-anchored transmembrane proteins [12]. Intriguingly, our sequence searches suggest that many other prokaryotic SecE orthologues are similar to that of *S. coelicolor* in that they appear to lack signal sequences and have a single, C-terminal transmembrane domain. For example, the SecE orthologues in all the sequences streptomycetes are all predicted to be shorter proteins, similar in length to that of SCO4646, and to have a single predicted transmembrane domain at their C-terminus. Remarkably, the SecE orthologue in the very well-studied model organism *Bacillus subtilis* (NCBI locus tag NP_387981) is also a shorter protein of 59 amino acid residues with a single, C-terminal transmembrane domain and no obvious N-terminal signal sequence. This appears also to be the case in the important pathogens *Staphylococcus aureus* (NCBI locus tag AAB54017) and *Enterococcus faecalis* (NCBI locus tag EEN75976), both of which are smaller proteins with one predicted C-terminal membrane spanning domain like that of *S. coelicolor*. The *M. tuberculosis* SecE protein is a longer protein of 161 amino acid residues however it too appears to lack a signal sequence and has a single, C-terminal transmembrane domain, unlike that of *E. coli.*

The article "Bacterial Transmembrane Proteins that Lack N-Terminal Signal Sequences" was published in 2011. Journal: PLoS One.

While we have identified this class of bacterial membrane proteins, the targeting apparatus and mechanism remains unknown. We have demonstrated that the C-terminal transmembrane domain is sufficient for localization; suggesting a targeting pathway that is independent of the SRP. Recent bioinformatics suggests that *Archea* and eukaryote TAMPs target via a similar set of machinery, the archeon ArsA and eukaryote equivalent the Get3 complex; however, the bacterial equivalent lacks key residues for membrane protein targeting, suggesting bacterial ArsA is not the TAMP targeting machinery [15]. The eukaryotic TAMPs are all predicted to insert their transmembrane domains into the membrane and sit facing their N-termini to the cytosol from either the mitochondrial outer membrane or the endoplasmic reticulum (N-terminus “in”) [31]. An interesting development in our analysis is the variation in predicted topology of the TAMPs from *S. coelicolor* (Table 1) with some facing the cytosol (N-terminus “in”) and some exterior to the cell (N-terminus “out”). Preliminary biochemical evidence has confirmed these 2 bacterial orientations (Figure 5). This requirement to cross the lipid bilayer may be the reason for a differing targeting mechanism for bacterial TAMPs in contrast to archeon and eukaryotes as translocation machinery may be required for proper translocation across the membrane. Based on known membrane targeting machinery, bacterial possibilities could include YidC as YidC is capable of targeting membrane proteins independent of the Sec translocon [8]. It has been previously reported that YidC alone is capable of inserting *E. coli* SecE, a SecE with multiple TMs, into the membrane [32]. Despite this possibility, YidC targeting of bacterial TAMPs has yet to be explored. The identification of a new targeting pathway could pose as an important target for an antimicrobial agent, especially in light of a potentially differing targeting pathway from eukaryotes.

The article "Bacterial Transmembrane Proteins that Lack N-Terminal Signal Sequences" was published in 2011. Journal: PLoS One.

## Materials and Methods

### Bioinformatics

The TAMP finder program was used as previously reported (Brito et al, Manuscript in Preparation). Transmembrane domains were detected using the TMHMM software available at http://www.cbs.dtu.dk/services/TMHMM/ and signal sequences were assessed using the SignalP software available online at http://www.cbs.dtu.dk/services/SignalP/. Hydrophilicity and hydrophobicity of the N-terminal regions was calculated using the online program http://www.innovagen.se/custom-peptide-synthesis/peptide-property-calculator/peptide-property-calculator.asp.

### Strains, plasmids and general growth conditions

*E. coli* strains were grown at 37°C in Luria broth medium. Plasmid construction was performed in *E. coli* strain XL1 blue (Stratagene); while *E. coli* strain ET12567 containing the pUZ8002 plasmid was used for conjugal transfer of plasmids into *S. coelicolor* [33]. *S. coelicolor* M145 was used to test the membrane protein predictions. *Streptomyces* strains were grown at 30°C on SFM agar for matings and R2YE for general restreaking. Liquid cultures of *S. coelicolor* were grown in R5 medium supplemented with 7% PEG-8000 [34]. Antibiotic concentrations were 50 µg/ml kanamycin, 50 µg/ml apramycin, 35 µg/ml chloramphenicol, 30 µg/ml thiostrepton and 25 µg/ml nalidixic acid.

### Construction of TAMP overexpression vectors

Putative membrane proteins SCO2900, SCO2973, SCO4008, SCO4646 and SCO7133 were amplified from *S. coelicolor* chromosomal DNA via PCR introducing a FLAG epitope (DYKDDDDK) at their N-termini for Western blot analysis, see Table 2 for primers. NdeI and BamHI restriction sites were introduced upstream and downstream of the genes, respectively, to allow for introduction into the *Streptomyces* overexpression vectors pIJ6902 and pIJ8600 [35], [36]. The cytoplasmic protein ActR was amplified in the same manner and introduced into pIJ6902.

**Table 2:** Primers used in this work.

Construct	Primer Name	Sequence 5′ to 3′
**FLAG-tag over-expression in pIJ6902**		
ActR	ActR-For	CATATGGACTACAAGGACGACGACGACAAGATGTCGCGAAGCGAGGAAGG
	ActR-Rev	GGCGTAGAGGATCCGAAGGC
SCO2900	2900-For	CATATGGACTACAAGGACGACGACGACAAGGTGGCGGACACGTCGGACAT
	2900-Rev	ATCCGGATCCGCAGCTTG
SCO2973	2973-For	CATATGGACTACAAGGACGACGACGACAAGTTGGCACGGAAGATCGGCAG
	2973-Rev	TCCAGCGTAACGGATCCGTC
SCO4646	4646-For	CATATGGACTACAAGGACGACGACGACAAGGTGACGGACGCCGTG
	4646-Rev	CGGGATCCTCGGCGCCCTTCG
SCO7133	7133-For	CATATGGACTACAAGGACGACGACGACAAGATGGACACGAGCAAGCAGGC
	7133-Rev	GCTACGGATCCCGCGGT
**FLAG-tag over-expression in pIJ8660**		
SCO4008	4008-For	CATATGGACTACAAGGACGACGACGACAAGATGGCAGCAAAGGACCCC
	4008-Rev	GGATCCTCACCGGTCGACGATGCG
**eGFP fusion of TM in pIJ6902**		
eGFP	eGFP-For	CGGCGGACATATGGTGAGCA
	eGFP-Rev	TCTTCTAGAGGTACGGGCTG
	eGFP*-Rev	GGCGGCCTCTAGACTTGTAC
eGFP-2973	eGFP2973-For	CCCGGCTCTAGACGCAACCG
	eGFP2973-Rev	CCGGGGATCCGTCCAGCGGT
eGFP-4646	eGFP4646-For	AGGTCGTCTGGTCTAGACGC
	eGFP4646-Rev	CTCGGTACCCGGGGATCCCC
eGFP-7133	eGFP7133-For	GCCGAGTCTAGACACCGACT
	eGFP7133-Rev	CTCGGTACCCGGGGATCCCG

The article "Bacterial Transmembrane Proteins that Lack N-Terminal Signal Sequences" was published in 2011. Journal: PLoS One.

### Construction of eGFP-tail anchor fusions

The eGFP gene was amplified from the plasmid pIJ8668, removing the stop codon and introducing an XbaI restriction site downstream for introduction into pIJ6902, see Table 2 for primers. The eGFP gene was also cloned in a similar manner but containing the stop codon for use as a cytoplasmic control (eGFP*-Rev primer). The putative tail anchor transmembrane domains from SCO2973, SCO4646 and SCO7133 were amplified including 11 residues upstream from the predicted transmembrane domain via PCR, introducing XbaI and BamHI for introduction downstream of the eGFP gene, primers are listed in Table 2.

### Separation of membrane and cytoplasmic fractions

*S. coelicolor* strains containing the TAMP overexpression vectors and the eGFP-tail anchor fusions were grown in liquid culture for 16 hours prior to induction. Cultures were induced for 45 min with 30 µg/ml thiostrepton. Cells were washed once with 10.3% sucrose and resupended in P buffer containing 2 mg/ml lysozyme [34]. Protoplasts were created by incubation at 30°C for 1 hour and harvested by filtering through cotton and centrifugation at 7,000×g for 10 min [34]. The pellet was resuspended in lysis buffer (150 mM Hepes pH 7.3, 150 mM NaCl, 3 mM DTT, 30% glycerol) with protease inhibitor cocktail. Subsequent steps were all performed at 4°C. Protoplasts were sonicated for 2 min at 5 sec intervals following 10 sec rest. The lysate was centrifuged at 7,000×g for 10 min and the supernatant was centrifuged at 100,000×g for 1 hr.

### Sucrose gradient ultracentrifugation

50 µg of total protein from the membrane fractions were loaded to the top of sucrose step gradients containing 60% sucrose (4 ml Tris pH 8), 40% sucrose (4 ml Tris pH 8) and 20% sucrose (3 ml Tris pH 8). Gradients were centrifuged at 100,000×g for 16 hr at 4°C and 1 ml fractions were collected by piercing a needle in the bottom of the centrifuge tube and collecting the flow through.

### Sodium carbonate extraction

Cell lysate was prepared as described above. The lysate was mixed on ice with an equal volume of 0.2 M sodium carbonate (pH 11.4) or 0.2 M sucrose (pH 7.8) and centrifuged at 4°C for 1 hr. Following centrifugation at 100,000×g, the supernatant was neutralized with glacial acetic acid and the pellet was resuspended in lysis buffer. The peripheral membrane protein RamC was used as a control for extraction by sodium carbonate. Preparation of lysate for this analysis was performed as previously described [24].

The article "Bacterial Transmembrane Proteins that Lack N-Terminal Signal Sequences" was published in 2011. Journal: PLoS One.

### Proteinase K Digestion

A concentration range of 0, 1, 10, 15, 20, 25, 50, 75, 100 µg/µl Proteinase K (Sigma) was added to protoplasts and incubated on ice for 10 minutes. Proteolysis was stopped by the addition protease inhibitors (Roche), followed by the addition of 3× SDS loading buffer and heated to 95°C for 10 minutes. The degree of Proteinase K digestion was visualized by Western blot analysis using the anti-FLAG antibody (Sigma).

### Visualization of subcellular localization

Western blot analysis was used to determine the localization patterns of the TAMPs and eGFP-tail anchor fusions. For detection of the TAMPs anti-FLAG (Sigma) was used at a concentration of 1∶10,000 and anti-eGFP (Invitrogen) was used at a concentration of 1∶2,500 for eGFP fusion proteins. Antibodies against RamC were used at a concentration of 1∶1,000.
